# Comparison of Single-Person Laparoscopic Appendectomy Using a Novel Brace-Assisted Camera Holding System and Conventional Laparoscopic Appendectomy: A Neural Network Algorithm Analysis

**DOI:** 10.1155/2022/5915670

**Published:** 2022-09-19

**Authors:** Nengyun Zhang, Yuanhong Li, Renou Zhou

**Affiliations:** Department of General Surgery, The Affliated People's Hospital of Ningbo University, Ningbo 315040, Zhejiang, China

## Abstract

**Background:**

Acute appendicitis represents one of the main causes of surgical emergencies. It can be approached as an open appendectomy or a laparoscopic appendectomy (LA). However, LA generally requires the cooperation of a surgeon and an assistant. This study aims to compare the safety and efficacy of the novel brace-assisted single-person laparoscopic appendectomy (BASPLA) with conventional laparoscopic appendectomy (CLA) in the treatment of patients diagnosed with acute appendicitis by neural network algorithm analysis.

**Methods:**

Between January 2020 and December 2021,a total of 120 adult patients with acute appendicitis were randomized to the BASPLA group (62 cases) and the CLA group (58 cases).The clinical data were compared between the two groups, including demographics, clinical characteristics, and outcomes.

**Results:**

There was no significant difference in patients' pain scores before operation (*p* = 0.68) and after operation (*p* = 0.81) and patient-reported cosmetic scores (*p* = 0.43) between the two groups. Operation time in the BASPLA group was longer than that in the CLA group (*p*<0.001). There were no significant differences in the conversion rate (*p* = 0.94), analgesics required before (*p* = 0.91) and after the operation (*p* = 0.78), intraoperative bleeding (*p* = 0.53), recovery of bowel movement time (*p* = 0.26), hospital stay (*p* = 0.06), and complication rate (*p* = 0.84) between the two groups.

**Conclusions:**

BASPLA for adult acute appendicitis can be a substitute for CLA, BASPLA is comparable to CLA in postoperative pain and quality of life. Compared to surgical assistants, it not only provides a stable, clear image for the surgeon but also frees up personnel. Especially in emergency surgery, it can achieve satisfactory clinical efficacy without requiring an assistant.

## 1. Introduction

The appendix is a tiny tubular structure at the end of the cecum, with many bacteria in the cavity. In this case, the faecalite, parasite or mesentery of the appendix is too short, the appendix will be distorted, resulting in the accumulation of secretions, increased internal pressure, and blood flow supply is blocked, so that the bacteria in the appendix cavity with the help of damaged mucosa invasion and inflammatory reaction. The appendiceal mucosa contains abundant lymphoid tissues and it can also block the appendix cavity after an enlarged submucosal lymphoid tissue. Congenital appendicular malformations and gastrointestinal dysfunction can also lead to appendix infections. After appendix infection, the pathological changes can be divided into acute simple appendicitis, acute suppurative appendicitis, gangrenous appendicitis, acute perforated appendicitis, and perituronal appendiceal abscess. Acute appendicitis is the most common acute abdominal disease in gastrointestinal surgery. Laparoscopic appendectomy (LA) has gradually become the gold standard for the surgical treatment of appendicitis [1]. At present, the traditional laparoscopic appendectomy (CLA) is basically a three-hole method, which needs to be completed together with a main surgeon and an assistant. However, since some patients with acute appendicitis were admitted at night and there were short of doctors on duty, the double-person mode can be hardly applied. At this time, a single-person laparoscopic appendectomy is particularly necessary. Referring to relevant literature, robot-assisted cameras in foreign countries have been reported [2], but the robot-assisted systems are expensive and difficult to implement in most hospitals in China. So, it is extremely necessary to find a simple and feasible brace-assisted camera holding system.

Appendicitis is an acute abdominal disease with a high incidence in clinical practice, and most patients with appendicitis need surgical resection. In laparoscopic surgery, the surgical incision is in direct contact with the trocar; the abdominal wall is swollen due to pneumoperitoneum; and the peritoneal exudate has less chance of contact with the surgical incision. When the appendix is removed from the abdominal cavity, it is protected by the specimen bag from direct contact with the surgical incision, reducing the incision infection rate. It is the most commonly used method for the treatment of appendix surgery.

In recent years, with the rapid development and popularity of laparoscopic technology, at the same time, due to the trauma of laparoscopic technology. A series of advantages, such as small, beautiful incisions, and quick postoperative recovery, have been widely used in the treatment of clinical appendicitis patients. In a conventional laparoscopic appendectomy, the patient's appendix needs to be removed through a trocar puncture hole, but it is relatively difficult to remove appendicitis patients with severe swelling. In addition, if the patient's mesangial edema and adhesion are more serious, usually accompanied by mesangial torsion, coupled with the relatively high difficulty of adjusting the operation angle during laparoscopic operation, forced separation of the patient's mesangial root is prone to bleeding.

An artificial neural network is an artificial intelligence method widely used in recent years to simulate the structure and function of the human brain nervous system. It adopts a nonlinear parallel processing mode and has strong learning and adaptation ability, which can be used to analyze influencing factors. A BP (backpropagation) neural network is a nonlinear uncertainty mathematical model and a multilayer feedforward artificial neural network with a continuous transfer function. Its training method is the error backpropagation algorithm (BP algorithm), and the weight and threshold of the network are constantly modified with the goal of minimizing mean square error, so as to finally fit data with high accuracy. The BP neural network has no requirements on the distribution of data, has a variety of connection functions, is not sensitive to the influence of multicollinearity and outliers, and can qualitative reveal the impact of input variables on output variables, so as to achieve the purpose of analyzing the influencing factors. Genetic algorithm (GA) is another artificial intelligence method to simulate biological evolution. It follows the principle of “survival of the fittest” and selects the best evolved individuals as the optimal solution. This method has the special point of global optimization, which can overcome the local optimization defect of the BP algorithm, optimize the initial weight and threshold value of the BP neural network, improve the stability of the BP neural network, and shorten the time. Conventional laparoscopic appendectomy (CLA) needs to be done together with the chief surgeon and assistant (Figure 1). However, because some patients with acute appendicitis are admitted at night and have insufficient doctors on duty, it is difficult to apply the two-person mode. At this point, a person undergoing a prosthetic appendectomy is particularly necessary. The new brace-assisted single-person laparoscopic appendectomy (BASPLA) is cheap and widespread and can also be used for other operations. This paper studies the effect of the new support-assisted single laparoscopic appendectomy (BASPLA) to explore a manpower-saving solution.

## 2. Materials and Methods

### 2.1. Case Selection

Acute appendicitis patients admitted to the General Surgery Department of the Affiliated People's Hospital of Ningbo University between January 2020 and December 2021 were included in this study. All included patients with a diagnosis of appendicitis met the following criteria [3–5].

1. Right lower abdominal pain or perumbilical pain, later focused on the right lower quadrant, associated or not with nausea and/or vomiting
2. Physical examination of right lower abdominal tenderness, which can be accompanied by rebound pain
3. Body temperature > 38 °C, or white blood cells > 10 × 10^9^/L
4. Ultrasound scan or CT confirm the diagnosis of appendicitis©
5. Patients aged from 18 to 50 years' of age

The exclusion criteria were as follows:

1. Symptoms for more than 3 days
2. Right lower abdominal mass on palpitation or computer tomography indicating right lower abdominal mass
3. Patient did not consent to a laparoscopic appendectomy
4. Additional patients with the following conditions were also excluded: history of cirrhosis and coagulation disorders, generalized peritonitis, shock upon admission, previous abdominal surgery, ascites, suspected or proven malignancy, contraindication to general anesthesia , inability to give informed consent, and pregnancy. Signed informed consent was obtained from all patients.

One hundred and twenty patients met the inclusion criteria and were included in this study. There were 62 and 58 patients in the BASPLA group and the CLA group, respectively, using randomized digital tables. The study protocol was approved by the ethical committee of The People's Hospital Affiliated to Ningbo University. The study was registered with (2020) Annual Ethics Review (Medical) No. (041). The diagnostic criteria were as follows:

1. With the clinical manifestations and signs of acute appendicitis;
2. Laboratory tests and B-ultrasound imaging examination to support acute appendicitis.

### 2.2. Surgical Method

Preoperative examination items: Before surgery, urgent blood type examination, blood routine, liver and kidney function, blood coagulation routine, urine routine, blood amylase, blood HCG, and other tests are required to further clarify the diagnosis and exclude other diseases. Preoperative notes: preoperative appendix surgery includes 8 hours of preoperative fasting, water prohibition for 4 hours, and providing the patient with an intravenous fluid supplement to correct electrolyte disorders, preoperative second-generation cephalosporin antibiotics against infection, analgesia, omeprazole acid suppression and stomach protection, and other symptomatic treatment.

#### 2.2.1. Preoperative Treatment

(1) Prepare the skin of the surgical area; (2) use of antibiotics: Administration of intravenous 1.5 g cefuroxime 30 minutes before the skin cut. All the operations were performed by three senior general surgeons with more than five years of experience in laparoscopic appendectomy.

#### 2.2.2. CLA Group

After general anesthesia was administered, the patient was in a supine position. A 10 mm incision was made on the umbilicus; a needle was punctured into the abdominal cavity, and carbon dioxide was inflated into the abdominal cavity to reach an intraabdominal pressure of 14 mmHg. The air-abdominal needle was removed, the abdominal cavity was punctured with a 10 mm sleeve needle, and the inner core was removed. The laparoscopic head was placed into a 10 mm trocar around the abdominal cavity to check for collateral injury and surrounding appendix. A disposable 12 mm trocar was inserted at the outer edge of the right rectus abdominis (approximately, 5 cm to the right side of the umbilicus) and a 5 mm trocar above the pubic combination (proximately 3-4 cm under the umbilicus), where the grip clamp was placed. When three trocars are inserted, the laparoscopic camera is held by the assistant.

The appendix was lifted with a separation clamp, and the mesoappendix was dissected by the electrocoagulation hook and ligated with a 10 mm hemlock after being free out of the appendicular artery. After being completely free of the whole appendix, the appendix was cut by double ligation with 10 mm or 12 mm hemlock according to the thickness of the appendix. After the appendix was removed with a removal bag, the abdominal cavity was washed, items were counted, and the incision was stitched.

#### 2.2.3. BASPLA Group

General anesthesia and the incisions were performed in the same method as that in the CLA group. A novel brace-assisted camera holding system was used (Figure 2).

First, the surgical cloth was spread on the moving cart, and then we put an auxiliary brace into a sterile plastic sleeve and fixed it on the cart. The laparoscope was positioned on the brace-assisted holding system. Because the cart is equipped with four universal wheels, it can be adjusted during the surgery. Furthermore, the brace has joints and is adjustable. Therefore, the camera was flexibly modified from different angles according to the requirements of the surgeon to gain the best view of the surgical field during the operation. The LA was performed by a single surgeon, and an assistant was spared. After the appendix was removed, careful observation of the abdominal cavity was done to determine that there was no bleeding. After the incisions were closed, the laparoscope was unfixed from the holding system.

Surgical discharge index: Patients can meet the following conditions:

1. Normal body temperature, no fever, and discomfort for three consecutive days
2. Review routine blood indicators are within the roughly normal range
3. No abdominal pain, abdominal distension, and discomfort
4. Intestinal function recovery, no obvious abnormality after eating
5. Surgical incision heal well, no swelling, induration, no blood, and exudation

### 2.3. Data Collection

The following preoperative variables were analyzed: age, sex, body mass index (BMI) [6, 7], anesthesiological risk, according to the scale of the American Society of Anesthesiologists (ASA) [8, 9] physical status classification system(Table 1). In order to better compare the safety and efficacy of BASPLA and CLA in clinical applications, the pain, visual simulation scoring method (visual analogue scale, VAS [10]), aesthetic score of patient's incision [11](patient-reported outcome, PRO [12]), and relevant perioperative variables were included in the outcome evaluation.

All the following data were collected:

1. Incision aesthetics score [11] (0–10 points): the patient had a self-evaluation at 3 months of postoperative follow-up, very dissatisfied with 0 points, and very satisfied with 10 points
2. VAS score [10]: preoperative score and 24 hours postoperative score
3. Analgesia use
4. Surgical time
5. Surgical conversion rate
6. Intraoperative bleeding amount
7. The recovery time of bowel movement
8. Incidence of complications hospital stay
9. Postoperative pathologic diagnosis (Table 2–5).

### 2.4. Statistical Analysis

Statistical analysis of the data was performed using the IBM SPSS 22 software. Measurement data are expressed as mean ± standard deviation (*x* ± *s*). Comparison of two-sample means was performed using a *t* test. Ordinal data were obtained using the Kruskal–Wallis H test in the nonparametric tests; count data are expressed as rate (%) with *χ*^2^ tests. The results of the hypothesis test are listed on the forest map. Heterogeneity was analyzed by the *χ*^2^ test. *P*<0.05 was considered a statistically significant difference.

Follow-up method: This article mainly records the postoperative adverse reactions of patients through telephone, WeChat, and outpatient follow-up. Understand the patient's satisfaction with the surgical incision. All data were recorded and analyzed using statistical tools.

## 3. Result

### 3.1. General Basic Clinical Characteristics of the Enrolled Patients

A total of 120 patients diagnosed with acute appendicitis were included, of which 58 were submitted to CLA and 62 to BASPLA. Preoperative data of the patients are demonstrated in (Table 1).

There were no statistically significant differences in two groups such as gender (*P* = 0.83), age (*P* = 0.88), BMI (*P* = 0.18), and ASA score (*p* = 0.77).

### 3.2. Neural Network Algorithm Analysis

The neural network algorithm is a common method mainly used in medical imaging diagnosis. It can process the noise in the CT images, making the image results more accurate and contributing to the medical diagnostic results. Based on the advantages of the neural network algorithm, this paper has used it to analyze the diagnosis and effect analysis of the new brace-assisted camera keeping system and the traditional laparoscopic appendectomy, which can be better differentiated.

The preprocessing is divided into three steps: grayscale, negative image, and histogram processing. The airspace enhancement result obtained by grayscale processing can be expressed as follows:

(1) $$\begin{array}{c} G\left(\overset{\wedge }{y}\right)=\left[\frac{EH}{\left(xy\right)}\right]\text{.} \end{array}$$

In formula (1), it respectively, represents the image before and after grayscale processing and are the processing functions of the image grayscale enhancement operation. Negative image processing is also known as inverse image processing. Assuming that the gray level range of the initial medical image grayscale processing result is [0, L-1], the negative image operation of the image is to transform [0, L-1] to [L-1, 0] through transformation. The specific transformation process can be expressed as follows:

(2) $$\begin{array}{c} h\left(x,y\right)=L-1-F\left(x,y\right)\text{.} \end{array}$$

In formula (2), it is the gray value of the point after reverse color processing and represents the gray value of the image after gray processing [8]. The purpose of image histogram processing is to enhance the contrast of medical images so as to highlight the effective information in medical images, that is, tumor information. The discrete function corresponding to the gray statistical histogram of a medical image is as follows:

(3) $$\begin{array}{c} \left.G\right)\;P^{\left(sk\right)}=\pm k_{{\begin{array}{c} =\\ n \end{array}}^{0,1,\cdots L-1}} \end{array}$$

In formula (3), it represents the k-level gray value of the image, while and respectively represent the number of pixels with gray value and the total number of pixels in the image. The medical image preprocessing is completed by grayscale, negative image, and histogram processing.

### 3.3. The Inclusion of RIM's Algorithm

Among RIM algorithms, the Network Assisted Cell Change (NACC) selection algorithm is directly related to how the RIM neighborhood is configured on the live network. It can be seen from the logical flow chart of the NACC selection algorithm that there is a key parameter, max No Cells Nacc Csfb, which represents the maximum number of NACC elements. Each NACC element corresponds to a cell. This cell means the cell information contained in the RRC Connection Release message triggered by CS Fallback as defined in 3GPPTS36.331(Figure 3 and 4).

### 3.4. Comparison of Surgical Efficacy Data

The data analyzed related to the pain and incision aesthetics during perioperative period are shown in (Table 2).

There was also no significant difference between the two groups as to the comparison of surgery-related indicators between the two patient groups in (Table 3).

No significant statistical difference was observed in the measures (conversion to open surgery *P* = 0.94, intraoperative bleeding *P* = 0.53, anal exhaust time *P* = 0.26, complication *P* = 0.84, hospital stay *P* = 0.06) except that the operation time in BASPLA was slightly longer than the CLA(*P*<0.001). Complications in both groups are shown in detail in (Table 4).

They include incision infection, abdominal infection, puncture hole bleeding, intestinal leakage, and postoperative intestinal obstruction. Intraabdominal abscess and pulmonary infection. Postoperative pathological diagnosis is shown in (Table 5).

## 4. Discussion

Currently, a large number of surgeries are performed by laparoscopy. Appendectomy is no exception, and although it is a surgical emergency, it has become one of the most commonly used laparoscopic procedures in general surgery in the world. LA was first reported by Semm [13] in 1983 and has become the gold standard for surgical treatment of acute and chronic appendicitis. In recent years, SPLA [14] (single-port laparoscopic appendectomy) has been developed; single-hole laparoscopic surgery is the insertion of a puncture device with multiple operating channels, through the operating channels inserting the surgical instrument, usually with a small incision above the navel. Preliminary studies have shown that the effectiveness and safety of SPLA are not statistically different compared with conventional LA, and that the SPLA is better than LA in terms of incision aesthetics, and even some scholars have even suggested that SPLA may replace LA as the preferred procedure for appendectomy [14]. However, a common feature of both LA and SPLA is the need for the main surgeon and assistant to complete an operation. Sometimes it is a waste of human resources and relatively simple surgery such as the appendectomy can be done by the surgeon alone. With the assistant of braces, 62 cases of LA have been successfully performed. There was no significant difference in observational indicators, except for the slightly prolonged operation time of BASPLA compared with CLA, which may be caused by installing the bracket and setting of the sterile lens sleeve.

Images are commonly used information carriers, and medical images provide an important and reliable basis for disease diagnosis, clinical treatment, and teaching and scientific research. However, due to the instability of medical imaging equipment, noise is inevitably introduced in medical images. Therefore, it is necessary to analyze the influence of the neural network algorithm to improve the accuracy of the diagnostic results. Most previous reports on SPLA and CLA were retrospective studies [15–17], and a few randomized controlled studies [4, 18] also mainly used clinical objective indicators as outcome indicators, lacking PRO [12]. PRO refers to the report of the patient's own health status, functional status, and treatment feelings. The PRO is collected through a standardized scale that provides much more information than a clinician or physiological measurements, thus making the judgment of clinical efficacy more comprehensive, true, and reliable. The 2013 CONSORT statement recommended PRO as one of the outcome indicators to be reported in randomized controlled studies [19].Two PRO measures were used in this study: VAS and patient incision aesthetics score. Statistics show that there is no significant difference between the BASPLA and CLA. On the premise of the same network structure and training parameters, the fitting data R2 of the BP neural network has a large variation. This is because MATLAB will randomly give the initial weights and thresholds of the network during each training, and different initial weights and thresholds will produce different training results. Some training results are better, while others are worse. A genetic algorithm optimized the initial weight and threshold value of the neural network, ruler 2 is more stable. The data fitting results show that the GA neural network has fewer iterative steps compared with the BP neural network and can achieve the preset goal faster. As the number of hidden layer neurons increases, the number of fitting data for BP neural networks and GA-BP neural networks reaches the preset target also increases. The main advantage of the neural networks is that they outperform almost any other machine learning algorithm. However, there are some downsides, and that is what you need to focus on. As I said earlier, whether or not you should use deep learning depends largely on the problem you need to solve. In cancer detection, for example, high performance is crucial because the better the performance, the more people can be treated. However, for some machine learning problems, traditional algorithms can provide better results.

## Figures and Tables

**Figure 1:** Conventional laparoscopic appendectomy (CLA) in the operation.

**Figure 2:** Simple and feasible brace-assisted camera holding system fixed on the cart.

**Figure 3:** RIM algorithm matrix distribution pattern, an example.

**Figure 4:** RIM algorithm matrix distribution pattern, another example.

**Table 1:** Preoperative data of patients.

Group	Sex (*n*)		Age	BMI (kg/m^2^)	ASA				
	M	F			I	II	III	IV	V
BASPLA (*n* = )	33	29	33.25 ± 11.43	24.15 ± 3.45	50	11	1	0	0
CLA (*n* = )	32	26	33.57 ± 11.55	23.27 ± 3.72	48	9	1	0	0
*T*/*H*/*χ*^2^	0.05		0.15	1.34	0.08				
*P*	0.83		0.88	0.18	0.77				

**Table 2:** Evaluation of pain and incision aesthetics before and after surgery.

Time	Group	Analgesia use (*n*(%))	VAS grade (score)	Evaluation of the incision aesthetics
Preoperative	BASPLA	22 (35.48%)	6.4 ± 2.6	—
	CLA	20 (34.48%)	6.2 ± 2.7	—
	*χ* ^2^	0.01	0.41	
	*P*	0.91	0.68	

Postoperative	BASPLA	13 (20.97%)	3.2 ± 2.2	7.6 ± 1.3
	CLA	11 (18.97%)	3.3 ± 2.3	7.4 ± 1.5
	*t*/*χ*^2^	0.07	0.24	0.78
	*P*	0.78	0.81	0.43

**Table 3:** Comparison of surgery-related indicators between the two patient groups.

Group	Number (*n*)	Operation time(min)	Conversion to open surgery (*n*(%))	Intraoperative bleeding (ml)	Anal exhaust time (h)	Complication (*n*(%))	Hospital stay (d)
BASPLA	62	76.4 ± 20.5	3 (4.84%)	10.5 ± 6.2	25.5 ± 4.2	6 (9.68%)	5.2 ± 1.8
CLA	58	62.3 ± 18.2	2 (3.45%)	9.8 ± 5.8	24.6 ± 4.5	5 (8.62%)	4.6 ± 1.6
*t*/*χ*^2^		3.97	0.006	0.64	1.13	0.04	1.92
*P*		<0.001	0.94	0.53	0.26	0.84	0.06

**Table 4:** Postoperative complications (in detail).

	LA		Total	95% CI P
	BASPLA	CLA		
Complication	6 (9.68%)	5 (8.62%)	11 (9.17%)	0.04 to 0.14 0.84
Incision infection	1	2	3	—
Abdominal infection	2	1	3	—
Puncture hole bleeding	0	1	0	—
Intestinal leakage	0	0	0	—
Postoperative intestinal	1	1	2	—
Obstruction				—
Intraabdominal abscess	1	0	1	—
Pulmonary infection	1	0	1	

**Table 5:** Postoperative pathological diagnosis.

	LA		Total (*n*(%))	95% CI
	BASPLA	CLA		
Acute simple appendicitis	8	10	18 (15.00%)	0.09–0.22
Acute suppurative appendicitis	42	38	80 (66.67%)	0.58–0.75
Gangrene and perforated appendicitis	10	9	19 (15.83%)	0.09–0.23
Periappendiceal abscess	2	1	3 (2.50%)	−0.03–0.05

## Data Availability

The data in the text are available to the corresponding author.
